# Intragastric exposure to titanium dioxide nanoparticles induced nephrotoxicity in mice, assessed by physiological and gene expression modifications

This article has been retracted.

**DOI:** 10.1186/1743-8977-10-4

**Published:** 2013-02-13

**Authors:** Suxin Gui, Xuezi Sang, Lei Zheng, Yuguan Ze, Xiaoyang Zhao, Lei Sheng, Qingqing Sun, Zhe Cheng, Jie Cheng, Renping Hu, Ling Wang, Fashui Hong, Meng Tang

**Affiliations:** 1 Medical College of Soochow University, Suzhou, 215123, China; 2 Key Laboratory of Environmental Medicine and Engineering, Ministry of Education, School of Public Health, Southeast University, Nanjing, 210009, China; 3 Jiangsu key Laboratory for Biomaterials and Devices, Southeast University, Nanjing, 210009, China

**Keywords:** Titanium dioxide nanoparticles, Nephrotoxicity, Oxidative stress, Gene-expressed profile, Mice

## Abstract

**Background:**

Numerous studies have demonstrated that titanium dioxide nanoparticles (TiO_2_ NPs) induced nephrotoxicity in animals. However, the nephrotoxic multiple molecular mechanisms are not clearly understood.

**Methods:**

Mice were exposed to 2.5, 5 and 10 mg/kg TiO_2_ NPs by intragastric administration for 90 consecutive days, and their growth, element distribution, and oxidative stress in kidney as well as kidney gene expression profile were investigated using whole-genome microarray analysis technique.

**Results:**

Our findings suggest that TiO_2_ NPs resulted in significant reduction of renal glomerulus number, apoptosis, infiltration of inflammatory cells, tissue necrosis or disorganization of renal tubules, coupled with decreased body weight, increased kidney indices, unbalance of element distribution, production of reactive oxygen species and peroxidation of lipid, protein and DNA in mouse kidney tissue. Furthermore, microarray analysis showed significant alterations in the expression of 1, 246 genes in the 10 mg/kg TiO_2_ NPs-exposed kidney. Of the genes altered, 1006 genes were associated with immune/inflammatory responses, apoptosis, biological processes, oxidative stress, ion transport, metabolic processes, the cell cycle, signal transduction, cell component, transcription, translation and cell differentiation, respectively. Specifically, the vital up-regulation of *Bcl6, Cfi* and *Cfd* caused immune/ inflammatory responses, the significant alterations of *Axud1, Cyp4a12a, Cyp4a12b, Cyp4a14,* and *Cyp2d9* expression resulted in severe oxidative stress, and great suppression of *Birc5*, *Crap2,* and *Tfrc* expression led to renal cell apoptosis.

**Conclusions:**

*Axud1, Bcl6, Cf1, Cfd, Cyp4a12a, Cyp4a12b, Cyp2d9, Birc5, Crap2,* and *Tfrc* may be potential biomarkers of kidney toxicity caused by TiO_2_ NPs exposure.

## Background

The dynamically development of the nanotechnolo-gy industry has led to the wide-scale production and application of nanomaterials. Among the various nanomaterials, customarily titanium dioxide nanoparticles (TiO_2_ NPs), owing to their high surface area to particle mass ratio and high reactivity, have been used as nontoxic, chemical inert and biocompatible pigment products or photocatalysts in cosmetics, pharmaceuticals and paint industries [1-7]. However, their attractive properties are the source of reservations. The potential human toxicity and environmental impact of TiO_2_ NPs have attracted considerable attention with their increased use in industrial applications.

Recently, published data indicated that the toxicity of TiO_2_ NPs. Liu et al. had found that TiO_2_ NPs were absorbed and accumulated in the liver, lungs, brain, lymph nodes, and red blood cells [8]. Park et al. observed that TiO_2_ NPs induced apoptosis and micronuclei formation in Syrian hamster embryo fibroblasts and increased the production of nitric oxide and hydrogen peroxide in human bronchial epithelial cells [9]. Furthermore, an *in vitro* study showed that high concentration of TiO_2_ NPs caused renal proximal cell death [10]. TiO_2_ NPs were also supposed to impair nephric functions and cause nephric inflammation, which through reactive oxygen species (ROS) accumulation to reveal its toxicity [11]. Our previous study also demonstrated that exposure to TiO_2_ NPs induced nephric inflammation and nephric cell necrosis [12]. We hypothesize that TiO_2_ NPs -induced kidney damages in mice may have special biomarkers of toxicity.

Newly, a large body of *in vivo* animal model studies have shown the toxicologic characteristics which cause striking changes of gene expression of some nanomaterials in kidney. For instance, curcumin treatment can alter the gene expression profile of kidney in mice on endotoxin-induced renal inflammation [13]. In addition, nanocopper can result in widespread renal proximal tubule necrosis and dramatically gene expression alterations in rat kidney [14]. Furthermore, a recent report found that proteins were differentially expressed in mouse kidney by exposure to TiO_2_ NPs [15]. However, the synergistic molecular mechanisms of multiple genes activated by TiO_2_ NP-induced renal toxicity in animals and humans remain unclear. In this study, mice were exposed to 2.5, 5 and 10 mg/kg body weight (bw) TiO_2_ NPs for 90 consecutive days, and their growth, element distribution, and oxidative stress as well as kidney gene expression profile were investigated. Our findings suggested that exposure to TiO_2_ NPs resulted in histopathological changes, apoptosis, oxidative stress, and impairment of element balance in kidney with increased TiO_2_ NPs doses. Furthermore, microarray analysis showed marked alterations in the expression of 1006 genes were associated with immune/inflammatory responses, apoptosis, biological processes, oxidative stress, metabolic processes, the cell cycle, transport, signal transduction, cell component, transcription, translation, and cell differentiation in the 10 mg/kg TiO_2_ NPs-exposed kidney. Therefore, the application of TiO_2_ NPs should be carried out cautiously.

## Results

### TiO_2_ NPs characteristic

XRD measurements show that TiO_2_ NPs exhibit the anatase structure (Figure 1), and the average grain size calculated from the broadening of the (101) XRD peak of anatase was roughly 5.5 nm using the Scherrer’s equation. TEM demonstrated that the average size of the particles of powder (Figure 2a) and nanoparticles which suspended in HPMC solvent after 12 h and 24 h incubation ranged from 5—6 nm, respectively (Figure 2b and c), which is consistent with the XRD results. The value of the sample surface area was generally smaller than the one estimated from the particle size, and it would seem that the aggregation of the particles may cause such a decline (Table 1). To investigate the dispersion and the stability of the suspensions of TiO_2_ NPs, we detected the aggregated size and the zeta potential of TiO_2_ NPs in HPMC. After the 12 h and 24 h incubation, the mean hydrodynamic diameter of TiO_2_ NPs in HPMC solvent ranged between 208 and 330 nm (mostly being 294 nm), as measured by DLS (Figure 3a and b), which indicates that the majority of TiO_2_ NPs were clustered and aggregated in solution. In addition, the zeta potential was 7.57 mV and 9.28 mV, respectively, and the particle characteristics for the TiO_2_ NPs used in this study are summarized in Table 1. The leakage of Ti^4+^ ions from 12 h, 24 h and 48 h incubation of TiO_2_ NPs in HPMC solvent after centrifugation was measured by ICP-MS. However, Ti^4+^ contents were not detected in filtrate, which are lower than the detection limit of 0.074 ng/mL (not listed). Therefore, these results suggested that the Ti^4+^ ions leakage from TiO_2_ NPs is limited in HPMC incubation.

**Figure 1:** **The (101) X-ray diffraction peak of anatase TiO**_**2 **_**NPs.** The average grain size was about 5 nm by calculation of Scherrer’s equation.

**Figure 2:** **Transmission electron microscope image of anatase TiO**_**2 **_**NPs particles.** (**a**) TiO_2_ NPs powder; (**b**) TiO_2_ NPs suspended in HPMC solvent after incubation for 12 h; (**c**) TiO_2_ NPs suspended in HPMC solvent after incubation for 24 h. TEM images showed that the sizes of the TiO_2_ NPs powder or suspended in HPMC solvent for 12 h, 24 h were distributed from 5 to 6 nm, respectively.

**Figure 3:** **Hydrodynamic diameter distribution of TiO**_**2 **_**NPs in HPMC solvent using DLS characterization.** (**a**) Incubation for 12 h; (**b**) Incubation for 24 h.

**Table 1:** **Characteristics of TiO**_**2 **_**NPs**

**Sample**	**Crystllite size (nm)**	**Phase**	**Surface area (m**^**2**^**/g)**	**Composition**	**Zeta potential**
TiO_2_ NPs	5.5	Anatase	174.8	Ti, O	7.57(a), 9.28(b)

(a) Zeta potential after the 12 h incubation in 0.05% w/v HPMC solvent; (b) Zeta potential after the 24 h incubation in 0.05% w/v HPMC solvent.

### Body weight, coefficient of kidney and titanium accumulation

Titanium accumulation, bw, and kidney indices of mice are listed in Table 2. As shown, an increased TiO_2_ NPs dose led to a gradual decrease in bw, whereas kidney indices and titanium content were significantly increased (*P* < 0.05), indicating growth inhibition and kidney damage in mice. These findings were confirmed by subsequent renal histological and ultrastructural observations and oxidative stress assays.

**Table 2:** **Body weight, coefficient of kidney and titanium accumulation in mice kidney by intragastric administration of TiO**_**2 **_**NPs for 90 consecutive days**

**Index**	**TiO**_**2 **_**NPs (mg/kg bw)**			
	**0**	**2.5**	**5**	**10**
Net increase of body weight (g)	22.55 ± 1.13a	17.59 ± 0.88b	14.22 ± 0.71c	12.05 ± 0.61d
Relative weight of kidney (mg/g)	10.07 ± 0.50a	11.58 ± 0.58b	13.31 ± 0.67c	15.69 ± 0.78d
Ti content (ng/g tissue)	Not detected	105 ± 5a	193 ± 10b	366 ± 18bc

Different letters indicate significant differences between groups (p < 0.05). Values represent means ± SEM(N = 10).

### Mineral element contents

The contents of mineral elements in kidney provide insight into how mineral elements in the kidneys of mice responded to treatment with TiO_2_ NPs. The mineral elements in the kidney, such as Ca, Na, K, Mg, Zn, Cu and Fe, were determined and listed in Table 3. It can be seen that with increased doses, TiO_2_ NPs exposure led to marked increased Ca, K, Mg, Zn, and Cu contents, whereas Na, and Fe contents decreased (P < 0.05, Table 3).

**Table 3:** **Accumulation of metal elements in mouse kidney by intragastric administration of TiO**_**2 **_**NPs for 90 consecutive days**

**TiO**_**2 **_**NPs (mg/kg bw)**	**Metal element contents (μg/g tissue)**						
	**Ca**	**Na**	**K**	**Mg**	**Zn**	**Cu**	**Fe**
0	1054 ± 53a	3540 ± 177a	2383 ± 119a	138 ± 7a	9.88 ± 0.49a	1.986 ± 0.10a	33.26 ± 1.66a
2.5	1259 ± 63b	3083 ± 154b	3039 ± 152b	159 ± 8b	18.72 ± 0.94b	5.69 ± 0.28b	17.16 ± 0.86b
5	1486 ± 74c	2772 ± 139c	3866 ± 193c	215 ± 11c	31.89 ± 1.59c	10.27 ± 0.51c	9.81 ± 0.49c
10	1823 ± 91cd	2511 ± 125d	4839 ± 242d	300 ± 15d	47.88 ± 2.39d	18.48 ± 0.92d	2.326 ± 0.12d

Different letters indicate significant differences between groups (p < 0.05). Values represent means ± SEM(N = 5).

### Histopathological evaluation of kidney

Figure 4 presents the histopathological changes of kidneys in mice treated by TiO_2_ NPs exposure for 90 consecutive days. Unexposed kidney did not suggest any histological changes (Figure 4a), while those exposed to increased TiO_2_ NPs concentrations exhibited severe pathological changes**,** including significant reduction of renal glomerulus number, apoptosis or vacuolization, infiltration of inflammatory cells, cell abscission on vessel wall as well as tissue necrosis or disorganization of the renal tubules (Figure 4b, c and d), respectively. In addition, we also observed significant black agglomerates in the 10 mg/kg bw TiO_2_ NPs exposed kidney (Figure4d). Confocal Raman microscopy further showed a characteristic TiO_2_ NPs peak in the black agglomerate (148 cm^-1^), which further confirmed the aggregation of TiO_2_ NPs in kidney (see the spectrum B in the Raman insets in Figure 4d). The results also suggested that exposure to TiO_2_ NPs deposited in the kidney and resulted in mouse renal injury.

**Figure 4:** **Histopathological observation of kidney caused by intragastric administration of TiO**_**2 **_**NPs for 90 consecutive days.** (**a**) Control, (**b**) 2.5 mg/kg TiO_2_ NPs, (**c**) 5 mg/kg TiO_2_ NPs, (**d**) 10 mg/kg TiO_2_ NPs. Yellow arrows indicate apoptosis or vacuolization, green arrows indicate cell abscission, fatty degeneration or cell necrosis, green virtual circle indicates infiltration of inflammatory cells, blue arrows indicate tissue necrosis or disorganization of renal tubules. Yellow virtual circle indicates TiO_2_ NPs aggregation. Arrow A spot is a representative cell that not engulfed the TiO_2_ NPs, while arrow B spot denotes a representative cell that loaded with TiO_2_ NPs. The right panels show the corresponding Raman spectra identifying the specific peaks at about 148 cm^-1^.

### Nephric ultrastructure evaluation

Changes to the nephric ultrastructure in mouse kidney are presented in Figure 5. As shown, the untreated mouse renal cells (control) contained round nucleus with homogeneous chromatin (Figure 5a), whereas with increased TiO_2_ NPs doses, the ultrastructure of renal cell from the TiO_2_ NPs-treated groups indicated a classical morphology characteristic of apoptosis, including mitochondria swelling, nuclear shrinkage, and chromatin marginalization in the renal cell (Figure 5b, c, and d). In addition, black deposits were also observed in the 10 mg/kg TiO_2_ NPs -exposed nephric cell via TEM (Figure 5d), Raman signals of TiO_2_ NPs was also exhibited via confocal Raman microscopy (Figure 5d).

**Figure 5:** **Ultrastructure of kidney in male mice caused by intragastric administration of TiO**_**2 **_**NPs for 90 consecutive days.** (**a**) Control, (**b**) 2.5 mg/kg TiO_2_ NPs, (**c**) 5 mg/kg TiO_2_ NPs, (**d**) 10 mg/kg TiO_2_ NPs. Yellow arrows indicate nucleus shrinkage, chromatin marginalization, green arrows indicate mitochondria swelling, and red arrows show presence of TiO_2_ NPs. Arrow A spot is a representative cell that not engulfed the TiO_2_ NPs, while arrow B spot denotes a representative cell that loaded with TiO_2_ NPs. The right panels show the corresponding Raman spectra identifying the specific peaks at about 148 cm^-1^.

### Oxidative stress

Alterations in ROS levels such as (

$$O_{2}^{–}$$

O_2_^**-**^ and H_2_O_2_) in the kidney can be regarded as markers of adaptive response of kidney to oxidative damage. As shown in Table 4, the levels of both

$$O_{2}^{–}$$

O_2_^**-**^ and H_2_O_2_ in mouse kidney following exposure to TiO_2_ NPs significantly increased compared with control values (P <0.05, Table 4). To prove the effects of TiO_2_ NPs on ROS generation, the levels of lipid peroxidation (MDA), protein peroxidation (carbonyl) and DNA peroxidation (8-OHdG) in mouse kidney were evaluated and presented in Table 4. The great increases of MDA, carbonyl and 8-OHdG in the TiO_2_ NPs -exposed kidney were also observed with increased TiO_2_ NPs doses (P < 0.05), suggesting that ROS accumulation led to lipid, protein, and DNA peroxidation in the kidney.

**Table 4:** **Oxidative stress in mouse kidney after intragastric administration of TiO**_**2 **_**NPs for 90 consecutive days**

**Oxidative stress**	**TiO**_**2 **_**NPs (mg/kg BW)**			
	**0**	**2.5**	**5**	**10**
O_2_^**.-**^ (nmol/mg prot. min)	18 ± 0.9a	25 ± 1.23b	38 ± 1.91c	43 ± 2.15d
H_2_O_2_ (nmol/mg prot. min)	31 ± 1.55a	46 ± 2.28b	77 ± 3.845c	92 ± 4.6d
MDA (μmol/ mg prot)	1.02 ± 0.05a	1.97 ± 0.10b	3.05 ± 0.15c	4.88 ± 0.24d
Carbonyl (μmol/mg prot)	0.51 ± 0.03a	1.13 ± 0.06b	1.89 ± 0.09c	2.79 ± 0.14d
8-OHdG (mg/g tissue)	0.48 ± 0.02a	2.16 ± 0.11b	3.58 ± 0.18c	5.87 ± 0.29d

Different letters indicate significant differences between groups (p < 0.05). Values represent means ± SEM (N = 5).

### Change in the gene expression profile

Treatment with high dose of 10 mg/kg bw of TiO_2_ NPs resulted in the most severe kidney damages, and these tissues were used to detect gene expression profiles to further explore the mechanisms of kidney damages induced by TiO_2_ NPs. Whole-genome expression profiling using mRNAs from pulmonary tissues of vehicle control groups and those treated with 10 mg/kg bw of TiO_2_ NPs exposed groups for 90 consecutive days were analyzed with the Illumina Bead Chip. Compared to the vehicle control group, 1, 246 genes of total genes (45, 000 genes) were found to be differentially expressed in the 10 mg/kg TiO_2_ NPs group (Additional file 1: Table S1), including 610 genes up-regulated and 636 down-regulated. Using the ontology-driven clustering algorithm included with the PANTHER Gene Expression Analysis Software (http://www.pantherdb.org/) as a tool for biological themes analysis, indicating that the 1, 006 genes among 1, 246 genes were associated with immune/inflammatory responses, apoptosis, biological processes, oxidative stress, metabolic processes, the cell cycle, ion transport, signal transduction, cell component, transcription, translation, and cell differentiation, another 240 genes function are unknown (Figure 6), respectively.

**Figure 6:** **Functional categorization of 1246 genes.** Genes were functionally classified based on the ontology-driven clustering approach of PANTHER.

### RT-PCR

To verify the accuracy of the microarray analysis, twenty-eight genes that demonstrated significantly different expression patterns were further evaluated by qRT-PCR due to their association with immune/inflammatory responses, apoptosis, oxidative stress, cell cycle, signal transduction and biological process. These 14 genes including Psmb5, Ngfrap1, Cycs, Tnfrsf12, Birc5, Fn1, Cd55, Cfi, Bub1b, Egr1, Nid1, Odc1, Cd34, and Apaf1 were up-regulated, whereas 14 genes including Bcl2l1, Ccl19, Ccl21a, Bmp6, Cd74, Cfd, Cxcl12, C3, Bcl6, Cygb, Klf1, Txnip, and Serpinalb were down-regulated (Table 5). The qRT-PCR analysis of all 28 genes displayed expression patterns comparable with the microarray data (i.e., either up- or down-regulation; Additional file 1: Table S1).

**Table 5:** RT-PCR validation of selected genes from microarray data

**Function**	**Gene**	**ΔΔCt**	**Fold**	**Microarray**
Apoptosis	Apaf1	0.516327	0.699149555	0.5535156
	Ngfrap1	0.15624	0.897360758	0.6713378
	Cycs	0.34444	0.787613639	0.7045653
	Tnfrsf12a	0.04954	0.966244365	0.655954
	Bcl2l1	-1.131909	2.191485298	1.663064
	Birc5	3.213009	0.107841995	0.10103
	Fn1	0.470814	0.721557364	0.4940369
	Ccl19	-2.490308	5.618978967	4.313047
	Ccl21a	-1.826821	3.547545038	2.850085
Immune/Inflammatory response	Bmp6	-1.291201	2.447317025	40.56928
	Cd55	0.54583	0.684997202	0.3824578
	Cd74	-1.327117	2.509007877	1.832029
	Cfd	-1.861094	3.632830363	2.601335
	Cfi	1.259912	0.417569429	0.3720603
	Cxcl12	-1.913449	3.76708608	2.043431
	C3	-1.580409	2.990546189	1.886813
	Cd34	0.282201	0.822335491	0.4588617
	Bcl6	-2.069258	4.196707749	3.073497
Oxidative stress	Cygb	-1.439087	2.711492162	1.646112
	Gpx7	0.585512	0.666412792	0.3389097
	Psmb5	0.057543	0.960899198	0.6914788
Cell cycle	Klf1	-1.646997	3.131810673	2.100916
	Bub1b	3.216187	0.1076047	0.2573011
	Txnip	-1.615053	3.063228525	1.648611
Signal transduction	Egr1	0.348792	0.785241322	0.5866718
	Nid1	0.918823	0.528940372	0.3838886
Biological process	Odc1	1.576015	0.335407069	0.3957967
	Serpinalb	-2.035634	4.100028676	3.299695

## Discussion

NPs were shown to attain the systemic circulation after ingestion, inhalation or intravenous injection. They can distribute to several organs like kidney, liver, spleen, heart, brain, and ovary [16-20]. The kidney has been known to eliminate harmful substances from the body, thus NPs assimilate in the systemic circulation can be filtered by renal clearance [21,22]. In this study, we found that intragastric administration of 2.5, 5, and 10 mg/kg bw of TiO_2_ NPs for 90 consecutive days induced bw reduction, increased kidney indices, TiO_2_ NPs deposition (Table 2), renal inflammation, tissue necrosis or disorganization of renal tubules (Figure 4), and renal apoptosis (Figure 5) in mouse kidney tissues coupled with element unbalance (Table 3), and severe oxidative stress, significant production of

$$O_{2}^{.–}$$

O_2_^**.**-^and H_2_O_2_, and peroxidation of lipids, proteins, and DNA (Table 4). The renal damages and oxidative stress following exposure to TiO_2_ NPs may be involved in impaired immune function and antioxidant capacity in mice and, thus, may be associated with changed gene expression in renal tissue. Large-scale gene expression analysis provides an approach to obtain a global view of the genomic changes and to gain insights into the detailed mechanisms behind the pathogenesis of various diseases [23]. To elucidate the molecular mechanisms of kidney damages and identify specific biomarkers induced by TiO_2_ NPs exposure, RNA microarray analysis of mouse kidney was performed to establish a global gene expression profile and identify toxicity-response genes in mice induced by exposure to 10 mg/kg bw of TiO_2_ NPs for 90 consecutive days. Our analysis indicated that the expression levels of 1, 246 genes were significantly changed and 1, 006 of these genes were involved in immune-inflammatory responses, oxidative stress, apoptosis, metabolism, the cell cycle, signal transduction, and ion transport etc. The main results are discussed below.

As we known, the development of kidney immune/nflammatory responses is result from the interaction between multifactor, multigene, multi-cell, multi-stage and inherent kidney cells, such as infiltration of inflammatory cells (Figure 4). The pathogenesis is involved in expression alterations of immune/inflammation-related genes. In this study, 36 genes linked to immune/inflammatory responses were significantly altered by exposure to 10 mg/kg TiO_2_ NPs (Figure 6). Of these genes altered, 29 genes were up-regulated and 7 genes were down-regulated. Ye et al. investigated that BCL-6 may regulate specific T-cell-mediated responses and can control germinal centre formation as a transcriptional switch. Modification of expression of BCL-6 in lymphoma results in the unnormal B cell proliferation and a deregulation of germinal centre formation [24], while B cell is an immune cell, so the up-regulated of the differentiation of B cell triggers the immune responses in the kidney. In our data, Bcl6 gene was greatly increased with a DiffScore of 67.89 in the kidney (Additional file 1: Table S1), suggesting that TiO_2_ NPs disordered the process of B cell differentiation, thus interfering with immune responses in mice. The inflammatory kidney disease membranoproliferative glomerulonephritis type II (MPGN2) is following the presence of complement C3. At the same time, complement factor I (cfi) can modulate the activation of C3 through the alternative pathway. And the breakdown of activated C3 is regulated by factor I, the deficiency of factor I causes uncontrolled C3 activation [25]. Our results showed that c3 gene up-regulated with a Diffscore of 30.23 and cfi gene down-regulated with a DiffScore of -54.62 following exposure to TiO_2_ NPs (Additional file 1: Table S1). The renal inflammation following exposure to TiO_2_ NPs was closely associated with overexpression of c3 gene and decreased expression of cfi gene in the kidney. While, our result also showed that complement factor D (Cfd) gene was observably up-regulated with a DiffScore of 52.09. Cfd is expressed in the kidney and plays a central role in the activation of the alternative pathway as a serine protease [26]. So the significant increased expression of Cfd gene demonstrated that TiO_2_ NPs exposure affected renal biochemical functions in the kidney [12]. CXCL12 (stromal cell-derived factor-1) is not only a unique homeostatic chemokine but also a potent small proinflammatory chemoattractant cytokines that binds primarily to CXC receptor 4 (CXCR4; CD184). As an inflammatory chemokine, CXCL12 has been immunodetected not only in normal tissues but also in many different inflammatory diseases [27]. In the present study, CXCL12 gene was up-regulated with a DiffScore of 28.02 after TiO_2_ NPs treatment, which was associated with infiltration of inflammatory cells in the kidney.

The current study suggested that TiO_2_ NPs exposure increased ROS significant production and led to peroxidation of lipids, proteins, and DNA in mouse renal tissue (Table 4), and caused renal cell apoptosis (Figure 5), which may be associated with alterations of oxidative stress-related or apoptosis-related gene expression. The overproduction of ROS has been shown to be closely associated with the induction of apoptotic and necrotic cell death in cell cultures [28]. This breaks down the balance of the oxidative/antioxidative system in the kidney, resulting in lipid peroxidation, which increased the permeability of mitochondrial membrane [11]. In our previous studies, TiO_2_ NPs were also shown to mediate apoptosis in the liver, spleen, brain, lung, and ovary in mice through the induction of ROS [21,29-35]. Meena et al. also showed that TiO_2_ NPs can induce oxidative stress which causes cell apoptosis in the kidney [36]. However, the apoptotic mechanism following TiO_2_ NPs -induced nephrotoxicity remains unclear. In the present study, our findings indicated that about 49 genes involved in oxidative stress and about 35 genes involved in apoptosis were dramatically altered in the 10 mg/kg TiO_2_ NPs exposed kidney, in which 49 were up-regulated and 35 were down-regulated (Figure 6). For example, Cyp4a12a, Cyp4a12b, Axud1, Ccl19, and Ccl21a genes were greatly up-regulated with DiffScores of 38.54, 123.6, 60.66, 83.27, and 28.86, respectively; while Cyp24a1, Akrlc18, Birc5, and E2F1 genes were significantly down-regulated with DiffScores of -33.79, -56.24, -101.23, and -66 (Additional file 1: Table S1), respectively. As we know, the cytochrome P450 (CYP) is a gene superfamily of enzymes encodes many isoforms and reveals a variety of catalytic activity, regulatory mechanisms and substrates [37]. Cyp4a12a, and Cyp4a12b are members of Cyp4 family of cytochrome P450 proteins and can hydroxylated arachidonic acid (AA) to 20-hydroxyeicosatetraenoic acid (20-HETE) effectively. Furthermore, Cyp4a12a and Cyp4a12b also effectively transformed eicosapentaenoic acid (EPA) into 19/20-OH- and 17, 18-epoxy-EPA, which are the predominant 20-HETE synthases in mouse kidney [38]. The up-regulation of Cyp4a12a and Cyp4a12b genes following exposure to TiO_2_ NPs illustrated that these abnormal expression may cause the disorder of oxidation-reduction process involved in 20-HETE production. The catabolic enzyme product of Cyp24a1 regulates the levels of hormonal 1, 25-dihydroxyvitamin D(3) (1, 25(OH)_2_D_3_) intracellular. The regulation of expression of this enzyme is crucial to the biological activity of 1, 25(OH)_2_D_3_[39]. Therefore, down-regulated of Cyp24a1 gene following exposure to TiO_2_ NPs suggested may disrupt the metabolism of 1, 25(OH)_2_D_3_ in the kidney_._ Aldo–keto reductases (AKRs) are members of a large enzymes family that catalyze NADPH- and NADH-dependent oxidoreduction of a wide variety of substrates, including 20α-Hydroxysteroid dehydrogenase (20α-HSD) simple carbohydrates and steroid hormones [40,41]. It is well-known that the AKR1C18 (20α-HSD) is a member of the AKR superfamily that catalyze the inactivation of progesterone, which stereoselective converts progesterone to its inactive metabolite 20α-hydroxy-4- pregnen-3-one (20α-HP) [40-43]. Down-regulation of Akrlc18 gene by TiO_2_ NPs exposure implied that TiO_2_ NPs may induce the activation of progesterone, which affects renal physiological processes. Axud1 (cysteine-serine-rich nuclear protein-1) also known as Csrnp-1 is an immediate early gene which strongly caused as a response to IL-2 in mouse T cells [44]. Overexpression of Axud1 conducts to apoptosis through the activation of the JNK pathway and inhibits mitosis [44]. In the study, significant increase of Axud1 gene expression caused by TiO_2_ NPs promoted renal cell apoptosis. Birc5 is a member of the inhibitor of apoptosis (IAP) gene family that encodes negative regulatory proteins which block apoptotic cell death. What’s more, the functions of Birc5 (survivin) are to enhance proliferation and survival of cells in the kidney [45]. Whereas, Birc5 gene down-regulation following exposure to TiO_2_ NPs may result in decreased survival of cells, and renal cells apoptosis in the kidney (Figure 5). It was previously reported that the stimulation of DCs with CCR7 ligands CCL19 and CCL21 inhibits well-known apoptotic hallmarks of serum-deprived DCs, including increased membrane blebs and membrane phosphatidylserine exposure, nuclear changes, and loss of mitochondria membrane potential [46]. In this study, we observed significant nucleus shrinkage, chromatin marginalization and mitochondria swelling in renal cell following exposure to TiO_2_ NPs (Figure 5). Ccl19 and Ccl21a upregulation, however, may serve as a protective role for kidney following TiO_2_ NPs-induced apoptosis. In addition, E2F1 is suggested to induce apoptosis and activation of p53-responsive target genes which coincides with an ability of E2F1 to induce accumulation of p53 protein. By affecting the accumulation of p53, E2F1 serves as a specific signal for the induction of apoptosis [47]. Decreased expression of E2F1 gene may also be associated with a protective role for kidney following TiO_2_ NPs–induced nephrotoxicity.

The equilibrium of various elements is essential for immune integrity in the kidney and plays an important role in renal physiology. Our data indicated that TiO_2_ NPs exposure led to significant increases in Ca, K, Mg, Zn, and Cu concentrations, but decreased Na, and Fe concentrations in the kidney (Table 3). The changes of these elements can provide useful information on physiology and pathology of kidney. To further clarify the molecular mechanisms of mineral element unbalance, we analyzed microarray data and found significant alterations of related-gene in the kidney. Sri gene overexpresses sorcin in K562 cells by gene transfection, which results in marked decrease of the level of cytosolic calcium and increased the ability of cell to resistance to apoptosis [48]. Intracellular Ca^2+^ homeostasis plays an important role in sustaining the biological functions of the cell and Ca^2+^overload may trigger apoptosis [49]. In contrast, our results showed that Sri gene was down-regulated with a Diffscore of -16.77 by TiO_2_ NPs exposure (Additional file 1: Table S1), which resulted in a significant Ca^2+^ overload in the kidney, thus leading to renal cell apoptosis. Slc10a6, also known as Soat, encodes protein of SOAT [50]. The transport conducted by SOAT is highly sodium dependence, indicating a symport transport with Na^+^ of the substrate [51]. In our data, Slc10a6 overexpressed with a Diffscore of 25.48, therefore, the increased Na^+^ concentration may be closely associated with Slc10a6 up-regulation in the kidney following exposure to TiO_2_ NPs. Establishing and maintaining high K^+^ and low Na^+^ in the cytoplasm are required for normal resting membrane potentials and various cellular activities. Therefore, the imbalance of Na^+^ and K^+^ caused by TiO_2_ NPs disturbed the ion homeostasis and cause a series of physiological disorders in the kidney. We also found that Cp gene was up-regulated with a Diffscore of 17.04, and Tfrc gene was dramatically down-regulated with a diffscore of -67.61 in the kidney (Additional file 1: Table S1). Ceruloplasmin (Cp), a copper-containing ferroxidase, is essential for body iron homeostasis as selective iron overburden takes place in aceruloplasminemia. Copper is an essential metal cofactor for numerous cuproenzymes which can catalyze some important biochemical reactions [52]. And the sticking point in the molecular mechanisms associated with copper-iron hypothesis is the cuproenzyme Cp [53]. Therefore, the increased Cu concentration and decreased Fe concentration may correlate with the up-regulation of Cp gene expression. In addition, Cu is a heavy metal, its overload following exposure to TiO_2_ NPs would lead to Cu poisoning in the kidney. Iron-restricted erythropoiesis is a common clinical condition in patients with chronic kidney disease. Iron status can be monitored by different parameters such as ferritin, transferrin saturation etc. Transferrin receptors (TfRc) are the principal pathway by which various organ cells to obtain iron for physiological requirements [54]. The number of TfRc on the cell surface displays the requirement of iron, so the synthesis of transferrin receptor is closely related to the iron requirements [55]. Decreased Fe level caused by TiO_2_ NPs may be also closely correlated to significant reduction of Tfrc gene expression, whereas Fe deficit would aggravate renal anemia and decrease immune capacity in the TiO_2_ NPs-exposed mice.

## Conclusions

The present study suggested that long-period exposure to TiO_2_ NPs resulted in severe kidney pathological changes and apoptosis, coupled with unbalance of mineral elements and severe oxidative stress. Furthermore, the nephrotoxicity following exposure to TiO_2_ NPs may be closely related to significant alterations in the expression of genes involved in immune/inflammatory responses, apoptosis, biological processes, oxidative stress, metabolic processes, the cell cycle, ion transport, signal transduction, cell component, transcription, translation, and cell differentiation. Axud1, Bcl6, Cf1, Cfd, Cyp4a12a, Cyp4a12b, Cyp2d9, Birc5, Crap2, and Tfrc genes may be potential biomarkers of kidney toxicity caused by TiO_2_ NPs exposure. Therefore, the application of TiO_2_ NPs in food, toothpastes, cosmetics and medicine should be carried out cautiously.

## Methods

### Preparation and characterization of TiO_2_ NPs

Nanoparticles anatase TiO_2_ was prepared via controlled hydrolysis of titanium tetrabutoxide. The details of the synthesis TiO_2_ NPs were previously described [34,56]. Briefly, colloidal titanium dioxide was prepared via a controlled hydrolysis of titanium tetrabutoxide. In a typical experiment, 1 mL of Ti (OC_4_H_9_)_4_ was dissolved in 20 mL of anhydrous isopropanol, and was added dropwise to 50 mL of double-distilled water that was adjusted to pH 1.5 with nitric acid under vigorous stirring at room temperature. The temperature of the solution was then raised to 60°C, and maintained for 6 h to promote better crystallization of TiO_2_ nanoparticles. Using a rotary evaporator, the resulting translucent colloidal suspension was evaporated yielding a nano-crystalline powder. The obtained powder was washed three times with isopropanol, and then dried at 50°C until the evaporation of the solvent was complete. A 0.5% w/v hydroxypropylmethylcellulose (HPMC) K4M was used as a suspending agent [57]. TiO_2_ powder was dispersed onto the surface of 0.5% w/v HPMC solution, and then the suspending solutions containing TiO_2_ particles were treated ultrasonically for 15–20 min and mechanically vibrated for 2 min or 3 min.

The particle sizes of both the powder and nanoparticles suspended in 0.5% w/v HPMC solution after incubation for 12 h and 24 h (5 mg/L) were determined using a TecnaiG220 transmission electron microscope (TEM) (FEI Co., USA) operating at 100 kV, respectively. In brief, particles were deposited in suspension onto carbon film TEM grids, and allowed to dry in air. The mean particle size was determined by measuring > 100 randomly sampled individual particles. X-ray-diffraction (XRD) patterns of TiO_2_ NPs were obtained at room temperature with a charge-coupled device (CCD) diffractometer (Mercury 3 Versatile CCD Detector; Rigaku Corporation, Tokyo, Japan) using Ni-filtered Cu Kα radiation. The surface area of each sample was determined by Brunauer–Emmett–Teller (BET) adsorption measurements on a Micromeritics ASAP 2020M + C instrument (Micromeritics Co., USA). The average aggregate or agglomerate size of the TiO_2_ NPs after incubation in 0.5% w/v HPMC solution for 12 h and 24 h (5 mg/L) was measured by dynamic light scattering (DLS) using a Zeta PALS + BI-90 Plus (Brookhaven Instruments Corp., USA) at a wavelength of 659 nm. The scattering angle was fixed at 90°. The Ti^4+^ ions leakage from TiO_2_ NPs at time 0 and/or after 12, 24, 48 h of incubation in 0.5% w/v HPMC was measured by Inductively coupled plasma-mass spectrometry (ICP-MS, Thermo Elemental X7, Thermo Electron Co., Finland) after sample was centrifugated at 1,719 × g for 10 min and filtrated with a 0.001 μm membrane filter.

### Animals and treatment

One hundred and twenty male CD-1 (Imprinting Control Region) mice aged 5 weeks with an average bw of 23 ± 2 g were purchased from the Animal Center of Soochow University (Jiangsu, China). All mice were housed in stainless steel cages in a ventilated animal facility with a temperature maintained at 24 ± 2°C and relative humidity of 60 ± 10% under a 12-h light/dark cycle. Distilled water and sterilized food were available *ad libitum*. Prior to dosing, the mice were acclimated to the environment for 5 days. All animals were handled in accordance with the guidelines and protocols approved by the Care and Use of Animals Committee of Soochow University (Jiangsu, China). All procedures used in the animal experiments conformed to the U.S. National Institutes of Health Guide for the Care and Use of Laboratory Animals [58].

An HPMC concentration of 0.5% was used as a suspending agent. TiO_2_ NPs powder was dispersed onto the surface of 0.5% w/v HPMC, and then the suspending solutions containing TiO_2_ NPs were treated ultrasonically for 30 min and mechanically vibrated for 5 min. For the experiment, the mice were randomly divided into four groups (N = 30 each), including a control group (treated with 0.5% w/v HPMC) and three experimental groups (treated with 2.5, 5, and 10 mg/kg bw TiO_2_ NPs, respectively). About the dose selection in this study, we consulted the report of World Health Organization in 1969. According to the report, LD50 of TiO_2_ for rats is larger than 12,000 mg/kg bw after oral administration. In addition, the quantity of TiO_2_ nanoparticles does not exceed 1% by weight of the food according to the Federal Regulations of US Government. The mice were weighed and then the TiO_2_ NPs suspensions were administered by intragastric administration every day for 90 days. All symptoms and deaths were carefully recorded daily. After the 90-day period, all mice were weighed, anesthetized with ether, and then sacrificed. Blood samples were collected from the eye vein by rapidly removing the eyeball and serum was collected by centrifuging the blood samples at 1, 200 × g for 10 min. The kidneys were quickly removed and placed on ice, and the kidneys were dissected and frozen at -80°C.

### Coefficient of kidney

After weighing the body and kidneys, the coefficients of kidney mass to bw were calculated as the ratio of kidney (wet weight, mg) to bw (g).

### Elemental content analysis

The frozen kidneys tissues were thawed and ~ 0.1 g samples were weighed, digested, and analyzed for titanium, sodium, magnesium, potassium, calcium, zinc, and iron content content. Briefly, prior to elemental analysis, the kidney tissues were digested overnight with nitric acid (ultrapure grade). After adding 0.5 mL of H_2_O_2_, the mixed solutions were incubated at 160°C in high-pressure reaction containers in an oven until the samples were completely digested. Then, the solutions were incubated at 120°C to remove any remaining nitric acid until the solutions were colorless and clear. Finally, the remaining solutions were diluted to 3 mL with 2% nitric acid. Inductively coupled plasma-mass spectrometry (Thermo Elemental X7; Thermo Electron Co., Waltham, MA, USA) was used to determine the titanium, sodium, magnesium, potassium, calcium, zinc, and iron concentration. Indium (20 ng/mL) was chosen as an internal standard element. Data are expressed as nanograms per gram fresh tissue.

### Histopathological evaluation of kidney

For pathological studies, all histopathological examinations were performed using standard laboratory procedures. The kidneys were embedded in paraffin blocks, then sliced (5-μm thickness), and placed on glass slides. After hematoxylin–eosin staining, the stained sections were evaluated by a histopathologist unaware of the treatments using light microscopy (U-III Multi-point Sensor System; Nikon, Tokyo, Japan).

### Observation of kidney ultastructure

The kidneys were fixed in fresh 0.1 M sodium cacodylate buffer containing 2.5% glutaraldehyde and 2% formaldehyde followed by a 2 h fixation period at 4°C with 1% osmium tetroxide in 50 mM sodium cacodylate (pH 7.2—7.4). Staining was performed overnight with 0.5% aqueous uranyl acetate, then the specimens were dehydrated in a graded series of ethanol (75, 85, 95, and 100%) and embedded in Epon 812 resin. Ultrathin sections were made, contrasted with uranyl acetate and lead citrate, and observed by TEM (model H600; Hitachi, Ltd., Tokyo, Japan). Kidney apoptosis was determined based on the changes in nuclear morphology (e.g., chromatin condensation and fragmentation).

### Confocal Raman microscopy of kidney sections

Raman analysis of renal glass or TEM slides was performed using backscattering geometry in a confocal configuration at room temperature in a HR-800 Raman microscope system equipped with a 632.817 nm HeNe laser (JY Co., France). It has been previously reported that when the size of TiO_2_ NPs reached to 6 nm, the Raman spectral peak was 148.7 cm^-1^[59]. Laser power and resolution were approximately 20 mW and 0.3 cm^-1^, respectively, while the integration time was adjusted to 1 s. The slides were scanned under the confocal Raman microscope.

### Oxidative stress assay

Superoxide ion (O_2_^·–^) in the kidney tissues was measured by monitoring the reduction of 3′-{1-[(phenylamino) carbonyl]-3, 4-tetrazolium}–bis (4-methoxy- 6-nitro) benzenesulfonic acid hydrate (XTT) in the presence of O_2_^**·–**^, as described by Oliveira et al. [60]. The detection of H_2_O_2_ in the kidney tissues was carried out by the xylenol orange assay [61].

Lipid peroxidation of kidneys was determined as the concentration of malondialdehyde (MDA) generated by the thiobarbituric acid (TBA) reaction as described by Buege and Aust [62]. Protein oxidation of kidneys was investigated according to the method of Fagan et al. by determining the carbonyl content [63]. DNA of kidneys was extracted using DNeasy Tissue Mini Kit (Nanjing Jiancheng Bioengineering Institute, Jiangsu, China) as described by the manufacturer. Formation of 8-OHdG was determined using the 8-OHdG ELISA kit (Japan Institute for the Control of Aging, Haruoka, Japan). This kit provides a competitive immunoassay for quantitative measurement of the oxidative DNA adduct 8-OHdG. It was carefully performed according to manufacturer’s instructions, and using a microplate varishaker-incubator, an automated microplate multi-reagent washer, and a computerized microplate reader.

### Microarray assay

Gene expression profiles of the kidney tissues isolated from 5 mice in the control and TiO_2_ NPs-treated groups were compared by microarray analysis using Illumina BeadChip technology (Illumina Inc., USA). Total RNA was isolated using the Ambion Illumina RNA Amplification Kit (cat no. 1755, Ambion, Inc., Austin, TX, USA) according to the manufacturer’s protocol, and stored at -80°C. RNA amplification is the standard method for preparing RNA samples for array analysis [64]. Total RNA was then submitted to Biostar Genechip, Inc. (Shanghai, China) to analyze RNA quality using a bioanalyzer and complementary RNA (cRNA) was generated and labeled using the one-cycle target labeling method. cRNA from each mouse was hybridized for 18 hrs at 55°C on Illumina HumanHT-12 v3.0 BeadChips, containing 45,200 probes (Illumina, Inc., San Diego, CA, USA), according to the manufacturer’sprotocolandsubsequently scanned with the Illumina BeadArray Reader 500. This program identifies differentially expressed genes and establishes the biological significance based on the Gene Ontology Consortium database (http://www.geneontology.org/GO.doc.html). Data analyses were performed with GenomeStudio software version 2009 (Illumina Inc., San Diego, CA, USA), by comparing all values obtained at each time point against the 0 hrs values. Data was normalized with the quantile normalization algorithm, and genes were considered as detected if the detection p-value was lower than 0.05. Statistical significance was calculated with the Illumina DiffScore, a proprietary algorithm that uses the bead standard deviation to build an error model. Only genes with a DiffScore ≤ -13 and ≥13, corresponding to a p-value of 0.05, were considered as statistical significant [65,66].

### Quantitative real-time PCR (qRT-PCR)

The levels of mRNA expression of *Apaf1, Bcl2l1, Bcl6, Bmp6, Birc5, Bub1b, C3, Ccl19, Ccl21a, Cd74, Odc1, Cd34, Cd55, Cfd, Cfi, Cxcl12, Cygb, Cycs, Egr1, Fn1 Klf1, Ngfrap1, Nid1, Psmb5, Serpinalb, Tnfrsf12, and Txnip* in the mouse kidney were determined using real-time quantitative RT polymerase chain reaction (RT-PCR) [67-69]. Synthesized complimentary DNA was generated by qRT-PCR with primers designed with Primer Express Software (Applied Biosystems, Foster City, CA, USA) according to the software guidelines, and PCR primer sequences are listed Table 6. The quantitative real-time PCR was performed by SYBR Green method using the special primers (as shown in Table 6) by the Applied Biosystems 7700 instrument (Applied Biosystems, USA).

**Table 6:** Real time PCR primer pairs

**Gene name**	**Description**	**Primer sequence**	**Primer size (bp)**
Refer-actin	Mactin-F	5^′^-GAGACCTTCAACACCCCAGC-3^′^	
	Mactin-R	5^′^-ATGTCACGCACGATTTCCC-3^′^	263
*Apaf1*	mApaf1-F	5'-TAGCGGCTCATCTGTTCTGTAG-3'	
	mApaf1-R	5'-CCACTTGAAGACAAAAGACCAA-3'	87
*Bcl2l1*	mBcl2l1-F	5'- ATTTCCCATCCCGCTGTG-3'	
	mBcl2l1-R	5'-GGCTAAAAGCACCTCACTCAAT-3'	82
*Bcl6*	mBcl6-F	5'- TTTCAATGATGGACGGGTGT-3'	
	mBcl6-R	5'- ACGCAGAATGTGGGAGGAGT-3'	118
*Birc5*	mBirc5-F	5'-TCTAAGCCACGCATCCCA-3'	
	mBirc5-R	5'-CAATAGAGCAAAGCCACAAAAC-3'	150
*Bmp6*	mBmp6-F	5'-ATTAAATATCCCTGGGTTGAAAGAC-3'	
	mBmp6-R	5'-CTGGGAATGGAACCTGAAAGAG-3'	117
*Bub1b*	mBub1b-F	5'-AATGGGTGGGGCTTTTGA-3'	
	mBub1b-R	5'-CCTGGCTGCTTGTCTTGC-3'	117
*C3*	mC3-F	5'-GGAGAAAAGCCCAACACCAG-3'	
	mC3-R	5'-GACAACCATAAACCACCATAGATTC-3'	148
*Ccl19*	mCcl19-F	5'-CCTCCTGATGCTCTGTCCCA-3'	
	mCcl19-R	5'-CGGTACCAAGCGGCTTTATT-3'	145
*Ccl21a*	mCcl21a-F	5'-CACGGTCCAACTCACAGGC-3'	
	mCcl21a-R	5'-TTGAAGCAGGGCAAGGGT-3'	102
*Cd34*	mCd34-F	5'-CTCAGTCCCCTGGCAGATTC-3'	
	mCd34-R	5'-GGACCCCTGTTCTCCCCTTA-3'	147
*Cd55*	mCd55-F	5'-AAATCCAGGAGACCAACCAAC-3'	
	mCd55-R	5'-CTGTAGATGTTCTTATTGGATGACG-3'	113
Cd74	Cd74-F	5'-ACGGCAAATGAAGTCAGAACA-3'	
	Cd74-R	5'-AAGACTACTAATGGGTCAGAAATGG-3'	97
*Cfd*	mCfd-F	5'-AGCAACCGCAGGGACACTT-3'	
	mCfd-R	5'-TTTGCCATTGCCACAGACG-3'	108
*Cfi*	Cfi-F	5'-CCCGAGTTCCCAGGTGTTTA-3'	
	Cfi-R	5'-GAAGGAGGTCATAGCTTCAGACA-3'	112
*Cxcl12*	mCxcl12-F	5'-CCAGTCAGCCTGAGCTACCG-3'	
	mCxcl12-R	5'-TTCTTCAGCCGTGCAACAA-3'	128
Cycs	mCycs-F	5'-CAACTCCGACTACAGCCACG-3'	
	mCycs-R	5'-GACACCACTATCACTCATTTCCCT-3'	134
*Cygb*	mCygb-F	5'-GCTCAGTGCCCTGCATTCC-3'	
	mCygb-R	5'-CCGTGGAGACCAGGTAGATGAC-3'	120
*Egr1*	mEgr1-F	5'-TTACCTACTGAGTAGGCTGCAGTT-3'	
	mEgr1-R	5'-GCAATAGAGCGCATTCAATGT-3'	141
*Fn1*	mFn1-F	5'-TGAAGCAACGTGCTATGACGA-3'	
	mFn1-R	5'-GTTCAGCAGCCCCAGGTCTAC-3'	149
*Klf1*	mKlf1-F	5'-ACCACCAGATAAATCAACTCAAATG-3'	
	mKlf1-R	5'-ATAGTAACGACAACAATCCTAGCAGA-3'	146
*Ngfrap1*	mNgfrap1-F	5'-GCCTTTAATGACCCGTTTGTG-3'	
	mNgfrap1-R	5'-TCCATGCTAATGGGCAACACT-3'	147
*Nid1*	mNid1-F	5'-ACCTCCTTTTCTTCTACTTTCACTG-3'	
	mNid1-R	5'-TCCAATTATTTAAGTAAAGACTCCCT-3'	122
*Odc1*	mOdc1-F	5'-TGCTGAGCAAGCGTTTGTAG-3'	
	mOdc1-R	5'-ATTCCCTGATGCCCAGTTATT-3'	107
*Psmb5*	mPsmb5-F	5'-GCTTCTGGGAGCGGTTGTT-3'	
	mPsmb5-R	5'-CATGTTAGCGAGCAGTTTGGA-3'	101
*Serpina1b*	mSerpina1b-F	5'-TGAGTCCACTGGGCATCAC-3'	
	mSerpina1b-R	5'-GCTTCTGTTCCTGTCTCATCG-3'	136
*Tnfrsf12a*	mTnfrsf12a-F	5'-CCAAGGACTGGGCTTAGAGTT-3'	
	mTnfrsf12a-R	5'-CCTTAGTATGGGTCGCTTTGTG-3'	114
*Txnip*	mTxnip-F	5'-CCTGGGTGACATTCTACATTGA-3'	
	mTxnip-R	5'-TAAGGCTTAGTGAGCTTCCGAG-3'	141

PCR primers used in the gene expression analysis.

### Statistical analysis

All results are expressed as means ± standard error of the mean(SEM). The significant differences were examined by unpaired Student's t-test using SPSS 19 software (USA). A p-value <0.05 was considered as statistically significant.

## Competing interests

The authors declare that they have no competing financial interests.

## Authors’ contributions

Conceived and designed the experiments: FH, MT, SG, XS, LZ, YZ, and XZ. Performed the experiments: FH, SG, XS, LZ, YZ, and XZ. Analyzed the data: FH, SG, XS, LZ, YZ, XZ, LS, QS, ZC, JC, RH, LW. Contributed reagents/materials/analysis tools: LS, QS, ZC, JC, RH, LW. Wrote the paper: FH, MT, SG, XS, LZ, YZ, and XZ. All authors read and approved the final manuscript.

## Supplementary Material

Additional file 1 Table S1 Genes which related to apoptosis, oxidative stress, immune/inflammatory, biological process, translation, cell differentiation, cell cycle, transcription, transport, metabolic process, cell component and signal transduction altered significantly by intragastric administration with TiO_2_ NPs for consecutive 3. Click here for file
